# Application of Montgomery T-Tube Placement in Treating Cotton-Myer IV Subglottic Airway Atresia after Bi-Level Airway Recanalization

**DOI:** 10.1155/2021/5517536

**Published:** 2021-05-20

**Authors:** Fengjie Wu, Yangwei Yao, Yangyang Gu, Meng Yang, Enguo Chen, Huihui Hu, Jisong Zhang, Liangliang Dong, Yeli Zhu

**Affiliations:** ^1^Department of Pulmonary and Critical Care Medicine, The Second Affiliated Hospital of Jiaxing University, Jiaxing, Zhejiang, China; ^2^Department of Pulmonary and Critical Care Medicine, Sir Run Run Shaw Hospital, College of Medicine, Zhejiang University, Hangzhou, Zhejiang, China; ^3^Department of the Operating Room, The Second Affiliated Hospital of Jiaxing University, Jiaxing, Zhejiang, China

## Abstract

**Objective:**

The purpose of this study is to explore the effectiveness and safety of Montgomery T-tube placement in treating Cotton-Myer IV subglottic airway atresia after bi-level airway recanalization.

**Methods:**

This study is a retrospective study. 11 patients who were treated for IV subglottic airway atresia between January 2017 and January 2019 in the Second Affiliated Hospital of Jiaxing University were involved in this study. The 11 patients all had undergone tracheotomies at our hospital, and they were transferred to the Department of Pulmonary and Critical Care Medicine for Montgomery T-tube placement after bi-level airway recanalization when their subglottic airway was atretic. Patients were observed for their clinical manifestations after placement. The effectiveness of T-tube placement after bi-level airway recanalization was assessed. The incidence of short-term and long-term complications after surgery was assessed. Patients were followed up for 3 to 24 months for evaluating their airway recovery.

**Results:**

T-tubes were successfully placed in 11 patients. The atretic airways of all patients were recanalized after treatment. Eight patients got restoration of vocal ability, and 3 patients could only say simple words. None of the patients needed assisted oxygen inhalation. The SpO2 average level was increased from 95 ± 2% before treatment to 97 ± 3% after treatment. Patients had significant relief of cough or sputum, and they had less difficulty in dyspnea. All short- or long-term complications were self-relieved or controlled without further malignant progression after treatment by doctors. The average postoperative extubating time was (14.86 ± 3.62) months.

**Conclusion:**

The application of Montgomery T-tube placement in treating Cotton-Myer IV subglottic airway atresia after bi-level airway recanalization is well effective and safe for patients, and it can be promoted in clinical treatment.

## 1. Introduction

Severe airway atresia can be life-threatening [1]. As a common complication after tracheotomy accompanied with cough, expectoration, and difficulty in breathing, subglottic airway stenosis occurs under the airway. Subglottic airway stenosis may influence the quality of patient's life, while severe stenosis may be life-threatening [2]. Subglottic airway stenosis can be classified into many kinds such as scarring airway stenosis. Scarring airway stenosis often occurs in patients who are easy to leave scars and undergo tracheotomy. Scars are formed at the site where the wound heals or where the physical injury on the airway occurs during surgery, resulting in airway stenosis [3]. Traditional treatments for airway stenosis involve surgical resection of the local airway where stenosis occurs [4]. However, in case of subglottic airway stenosis, the specificity of the occurrence site makes the traditional surgical resection difficult. Hence, for subglottic airway stenosis, a different treatment is needed.

One or more complication is prone to occur both during and after the treatment of airway stenosis [5]. A previous study showed that the length of airway resected in surgery may serve as a predictor of complications. When the length was longer than 4 cm, the incidence of complications showed a statistical difference, indicating that airway resection by surgery to treat airway stenosis is prone to induce the incidence of complications [6]. In addition, in the treatment of malignant airway stenosis with silicone Y stents, stent edge granulation tissue development occurred as early as in the first month after surgery, leading to early removal of the stents, which affected the treatment efficacy [7]. Furthermore, although silicone stents are less irritating to local tissues and relatively easy to remove, the tension of silicone stents is too low to be stable [7]. Thus, a new clinical treatment approach needs to be developed for airway stenosis.

There are studies on the use of Montgomery T-tube for treatment of airway stenosis. One study on treatment of the main type of airway stenosis by T-tubes showed that T-tubes could be placed at a high success rate and all patients had improvements in respiratory function and status, especially in the restoration of vocal ability. Besides, no serious postoperative complications were observed and no patients died from complications, demonstrating the feasibility and safety of the T-tube placement in the treatment of airway stenosis [8]. While for subglottic Cotton-Myer IV airway atresia, the use and efficacy of T-tubes are not clear.

This study investigates the effectiveness and safety of Montgomery T-tube placement after bi-level airway recanalization in the treatment of Cotton-Myer IV subglottic airway atresia after tracheotomy.

## 2. Methods

### 2.1. Experimental Design and Baseline Level

This study was a retrospective study. 11 patients who were treated for IV subglottic airway atresia between January 2017 and January 2019 in the Second Affiliated Hospital of Jiaxing University were involved in this study. All the patients had undergone tracheotomy in our hospital or other hospitals, and they were diagnosed as posttracheotomy Cotton-Myer IV subglottic airway atresia by CT (computed tomography) scanning and bronchoscopy. They accepted Montgomery T-tube (Boston Medical Products, USA) placement after bi-level airway recanalization at our hospital. The average age of the 11 patients was 48.05 ± 9.30. There were 4 male patients and 7 female patients. Patient's basic information about age, gender, the number of patients with preoperative oxygen inhalation, etc. was listed in Table 1.

### 2.2. Processes of T-Tube Placement

#### 2.2.1. Preparation

Patients were introduced to the surgery and asked to sign written informed consent. Routine examinations, including coagulation and electrocardiogram, were performed to exclude any contraindications to surgery. All patients were reexamined by CT scanning and bronchoscopy, while some patients had MRI (magnetic resonance imaging) reconstruction. The occurrence site, type, and length of airway stenosis of each patient were assessed. All patients were asked to undergo over 8 h of food and liquid fasting. Patients were provided with 2% lidocaine by aerosol inhalation for anesthesia 20 min before surgery to reduce airway reactivity. After total intravenous anesthesia, tracheostomy cannula was removed and replaced with a 6#–7# plastic tracheal cannula. Ventilators were connected for assisted inhalation.

#### 2.2.2. Bi-Level Recanalization

All the patients were kept horizontal and reclining during the operation. A STORZ rigid bronchoscope was inserted near the glottis under the guidance of a fiber bronchoscope. Then, an endotherm knife and rigid endoscope forceps were used for airway recanalization by means of gradually ablating the atretic airway to the distal end using blunt dissection technique. Meanwhile, vessel forceps and electrotome were used to gradually separate the atretic airway from the incision at distal glottis in a retrograde way. When the airway was recanalized, it was mechanically expanded with the rigid endoscope according to patient's situation for T-tube placement. Endotherm knife and rigid endoscope forceps were used to ablate and excise the granulation tissue from the inner wall of the airway.

#### 2.2.3. T-Tube Placement

According to the results of CT scan and bronchoscopy, a T-tube with a proper diameter was selected for each patient (Table 2) and the branch of the T-tube near the glottis was trimmed according to patient's own condition. The plastic trachea cannula was removed, and the branch of the T-tube at the distal glottis was inserted into the airway to the distal end. Meanwhile, the direction of the T-tube was adjusted by rigid forceps at the distal glottis. When the T-tube was placed in the airway completely, it was fixed and the wound was sutured. During the placement, the expansion of the T-tube should be noticed all the time.

#### 2.2.4. Postoperative Short-Term Care

One week after the T-tube placement, patients were given liquid budesonide and acetylcysteine by aerosol inhalation for anti-inflammation. Sputum retained in the T-tube was absorbed to prevent retention at the edge of the T-tube, which may affect patient's breathing. The clinical manifestations of the incision were carefully observed and the wound dressing was changed according to the situation.

### 2.3. Evaluation

The success rate of T-tube placement after bi-level airway recanalization was evaluated. Patient's clinical manifestations after the T-tube placement were observed. The effectiveness of the T-tube placement in the treatment of subglottic airway stenosis was assessed by calculating the proportion of the patients who required oxygen inhalation and comparing several indicators like SpO2 before and after treatment. Following the Modified Medical Research Council (mMRC) dyspnea scale [9], dyspnea is graded into 4 levels: grade 0—patients with obvious dyspnea symptoms, unable to leave the room, or shortness of breath during dressing and undressing; grade 1—patients must rest after walking on a flat ground for a few minutes or a distance of 100 m; grade 2—compared with peers, patients walk slowly due to breathing difficulties or resting necessity while walking on a flat ground; grade 3—patients who have shortness of breath during fast walking and walking uphill; and grade 4—no obvious breathing difficulty symptoms unless patients perform strenuous exercise. Meanwhile, postoperative complications were recorded.

### 2.4. Follow-Up Visit

Patients were followed up for 3 to 24 months after surgery. A total of 10 patients were involved in the whole follow-up period and 1 patient was lost to follow-up, with a follow-up rate of 90.9%. During the follow-up, chest CT, bronchoscopy, and other related examinations were performed on the patients to assess the airway recovery. Patient's extubating time was recorded.

### 2.5. Statistical Analysis

All data were statistically analyzed with SPSS 19.0 and the measurement data were presented with mean ± SD. *t*-test was used to analyze the paired data, and the numeration data were presented with %. Chi-square test or Fisher exact test was used to analyze enumeration data. *p* < 0.05 meant that data were statistically different.

## 3. Results

### 3.1. The Success Rate and Effectiveness of T-Tube Placement in Treatment of Subglottic Airway Stenosis

All 11 patients had successful T-tube placement and 5 of them had significantly relieved cough or expectoration. 5 of them had breathing difficulty before surgery, which was improved after surgery. During the surgery, there was no serious bleeding event. All 11 bleeding events were assessed as minor bleeding.

Indexes such as patient's autonomous respiration and SpO2 were assessed 7 days after surgery, and the results were listed in Table 3. Before T-tube placement, 8 patients needed assisted oxygen inhalation to release breathing difficulty. After treatment, oxygen inhalation was no longer necessary and 8 patients got restoration of vocal ability and 3 patients could only say simple words. Before surgery, the SpO2 of patients was 95 ± 2%, compared with 97 ± 3% after surgery. 10 patients had cough or expectoration before surgery while they got much better after surgery, and only 1 patient (9.1%) needed airway moistening by aerosol inhalation for sputum dilution. Before surgery, there was 1 patient (9.1%) assessed as grade 3 dyspnea and 1 patient (9.1%) as grade 4 dyspnea. After surgery, the dyspnea grade of the two patients was decreased to 1 or 2. Four patients (36.4%) were assessed as grade 1 dyspnea and 1 patient (9.1%) was of grade 2. These results demonstrated that T-tube placement was significantly effective in the treatment of subglottic airway atresia.

### 3.2. Safety of the T-Tube Placement in the Treatment of Subglottic Airway Stenosis

As listed in Table 4. regarding short-term complications, 1 patient (9.1%) had grade 2 mediastinal emphysema, 5 patients (45.5%) had grade 1 vocal cord edema, 1 patient (9.1%) had grade 1 hemoptysis, 2 patients (18.2%) had grade 1 bronchospasm, and 1 patient (9.1%) had grade 1 atrial fibrillation. Long-term complications were mainly sputum retention in T-tube and infection. 1 patient (9.1%) had sputum retention in the T-tube, 1 patient (9.1%) had lower respiratory infection, 3 patients (27.3%) had granulation tissue hyperplasia on the edge of the T-tube, 3 patients (27.3%) had a T-tube shift during the follow-up period after surgery and the T-tube needed to be replaced, and 2 patients (18.2%) had subcutaneous soft tissue infection. All short- or long-term complications were self-reduced or controlled by doctor's medical treatment without any malignant progression. The results of assessment at the short- or long-term complications after surgery demonstrated that T-tube placement in the treatment of subglottic airway stenosis was safe for patients.

### 3.3. Airway Recovery after Surgery

All patients were followed up after surgery for 3 to 24 months. One patient was lost to follow-up. The follow-up recorded the patient's extubating time. Only 2 patients were considered to be ready for extubating one year after surgery, and the 1-year extubating rate was 20.00%. All patients could remove the tubes two years after surgery and the two-year extubating rate was 100%. The average extubating time of patients was (14.86 ± 3.62) months, indicating that most patients needed at least 1 year of postoperative recovery before extubating.

## 4. Discussion

In clinical diagnosis, a patient is diagnosed with congenital subglottic stenosis when his cricoid cartilage region in the airway is stenosed in the condition of the patient never receiving endotracheal intubation [10]. However, iatrogenic subglottic stenosis is more common in clinical practice. Some surgeries, such as tracheostomy near the glottis, cricothyroidotomy, long-term intubation, and displacement of the tube in the airway, are all potential risks for subglottic stenosis [11]. A previous study used partial cricotracheal resection (PCTR) or extended cricotracheal resection (ECTR) to treat subglottic stenosis, but the surgery caused unilateral arytenoid prolapse in one patient, which severely affected the patient's life. Moreover, the patients should recover for a long time, with a median of 11 months after surgery [12]. Hence, surgical resection of the stenosed airway is not an optimal choice for treatment of subglottic stenosis. In contrast, there is a study analyzing the curative effect of T-tube placement on treating scarring stenosis of the cervical airway. The result showed that all the 37 patients underwent T-tube placement the first time in treating airway stenosis and the treatment period was at least 10 months, with an extubating rate of 83.7%, demonstrating the effectiveness of T-tube placement in treating cervical airway stenosis [13]. Furthermore, an experiment induced subglottic stenosis in animal models, and its results showed that endoscopic intervention treatment for subglottic stenosis is well instructive [14], which is of guiding significance for future intervention treatment with endoscopy for airway stenosis. Our study was targeted to patients with Cotton-Myer IV subglottic airway stenosis and retrospectively explored the effectiveness and safety of T-tube placement in treating subglottic airway stenosis with a rigid bronchoscope after bi-level airway recanalization.

It is useful and effective for T-tube placement in treating airway stenosis. T-tubes are left in the airway as a support after tracheotomy, maintaining airway patency. One case report showed that it was effective for a 12-year-old boy diagnosed with laryngeal airway stenosis to be treated with a 10 mm T-tube [15]. Consistently, our study showed that the T-tube placement was effective in treating subglottic airway atresia as well. Our findings showed that all patients did not need assisted oxygen inhalation anymore after surgery and the average SpO2 after surgery was raised. The results show statistical differences, indicating the significant efficacy of the T-tube placement in the treatment of subglottic airway stenosis. Meanwhile, the success rate and safety of T-tube placement are high. In a retrospective study, 20 patients who underwent the treatment of secondary benign airway stenosis after tracheotomy were successfully placed with a T-tube [16]. As such, 11 patients in this study were also successfully placed with T-tubes. Postoperative complications are classified into early complications and long-term complications. Early complications are mainly related to surgery [17], including postoperative fever, bleeding, mucus secretion, irritating cough, and short-term breathing difficulties, which can usually be relieved. The long-term complications are mainly the granulation tissue formation at the edge of the T-tube, the obstruction of the T-tube caused by the difficulty of expectoration, and secondary infection. The granulation tissue formation at the edge of the T-tube mainly occurs on the upper edge, which may be caused by the patient swallowing or speaking leading to the displacement of the T-tube, resulting in an excessive friction between the T-tube and the lumen mucosa, thereby stimulating granulation tissue formation [18]. A previous study also demonstrated that the most common complication that occurred after T-tube placement in treating laryngeal airway stenosis was granulation tissue formation [19]. In this study, the most common short-term complication that occurred was vocal cord edema, while the most common long-term complication that occurred was granulation tissue hyperplasia on the edge of the T-tube, which was similar to the results of the previous study. For the use of surgical resection for airway stenosis, relevant studies have shown that convalescence is long. For example, Wu et al. [20] suggested that the T-tube should be removed or replaced according to the situation after the T-tube is placed for 6 to 12 months. Our study had similar results from our postoperative follow-up that patients needed at least one year of postoperative recovery before T-tube removal. However, due to the small sample size of patients, the recovery time after the T-tube placement in treating subglottic airway atresia needs to be further discussed.

In conclusion, it is effective and safe to use Montgomery T-tube placement in treating Cotton-Myer IV subglottic airway atresia after bi-level airway recanalization and T-tube placement can be widely used in clinical treatment.

## Figures and Tables

**Table 1:** Baseline information of patients before T-tube placement.

Characteristics	Value (*N* = 11)
Age (years)	48.05 ± 9.30
Gender (%)	
Male	4 (36.4)
Female	7 (63.6)
Underlying disease (%)	
Cerebral hemorrhage	1 (9.09)
Craniocerebral trauma	1 (9.09)
Traffic accident trauma	3 (27.3)
Electric injury	2 (18.2)
Cerebral infarction	2 (18.2)
Granulomatous polyangiitis	2 (18.2)
Clinical symptoms (%)	
Aphasia	10 (90.9)
Cough	4 (36.4)
Expectoration	6 (54.5)
Dyspnea	5 (45.5)
Stenosis types (%)	
Granulation tissue development	5 (45.5)
Scarring stenosis	6 (54.5)
Tracheal wall atrophy	7 (63.6)
Tracheal distortion	6 (54.5)
Airway stenosis length (%)	
1 ~ 2 cm	2 (18.2)
2 ~ 3 cm	6 (54.5)
>3 cm	3 (27.3)

Multiple clinical symptoms and stenosis types of patients were complicated. SpO2: blood oxygen saturation.

**Table 2:** Sizes of T-tubes and operation processes.

Sizes of T-tubes and operation processes	*N* (%)
T-tube diameter	12 mm: 1 (9.1)
	13 mm: 5 (45.5)
	14 mm: 5 (45.5)

Mechanical expansion with rigid bronchoscope	11 (100)

Granulation tissue excision	10 (90.9)

Retrogradely tracheal blunt dissection	11 (100)

**Table 3:** Indexes of patients before and after surgery.

Index	Before	After	*p* value
Oxygen inhalation (%)			0.001
Yes	8 (72.7)	0 (0.0)	
No	3 (27.3)	11 (100)	
SpO2 (%)	95 ± 2	97 ± 3	0.049
Cough or expectoration (%)	10 (90.9)	1 (9.1)	0.003
Breathing difficulty (%)			0.444
Grade 1	1 (9.1)	4 (36.4)	
Grade 2	2 (18.2)	1 (9.1)	
Grade 3	1 (9.1)	0 (0.0)	
Grade 4	1 (9.1)	0 (0.0)	

**Table 4:** Short- or long-term complications after T-tube placement.

Complication	Occurrence rate (%), *N* = 11	Grade
Short term (<24 h)		
Mediastinal emphysema	1 (9.1)	2
Vocal cords edema	5 (45.5)	1
Hemoptysis	1 (9.1)	1
Bronchospasm	2 (18.2)	1
Atrial fibrillation	1 (9.1)	1
Long-term (>24 h)		
Sputum retention in T-tube	1 (9.1)	—
Lower respiratory infection	1 (9.1)	—
Granulation tissue hyperplasia on the edge of T-tube	3 (27.3)	—
T-tube replacement	3 (27.3)	—
Subcutaneous soft tissue infection	2 (18.2)	—

## Data Availability

The data used to support the findings of this study are included within the article. The data and materials in the current study are available from the corresponding author upon reasonable request.
